# Clinical Study on Different Methods of Internal Fixation for Treatment of Lisfranc Joint Injury

**DOI:** 10.1155/2021/1300920

**Published:** 2021-10-18

**Authors:** Songtao Jin, Lei Wang, Shiwei Zhou

**Affiliations:** ^1^Department of Orthopedics, Shaoxing People's Hospital, Shaoxing, Zhejiang 312000, China; ^2^Department of Emergency, Shaoxing People's Hospital, Shaoxing, Zhejiang 312000, China

## Abstract

The Lisfranc joints are mainly used to connect the forefoot and midfoot and maintain the stability of the arch of the foot. It is an important part of the arch of the foot. If the Lisfranc joints injury is not treated in time, it will cause poor walking, pain in the back of the foot, and even deformity or disability of the forefoot. The common treatment method is to select the Kirschner wires, screws, or steel plates for incisional repositioning internal fixation surgery. In our study, we used different materials to perform fixation surgery on Lisfranc joint injury patients. We measured the joint recovery, pain condition, complications, and biomechanical indexes of different groups of patients after the operation. The results of the study showed that compared with Kirschner wire and screw internal fixation, the use of shaped arch bridge-type microsteel plate internal fixation for the treatment of metatarsotarsal joint injury patients has better foot function recovery, fewer complications, and more reliable biomechanical strength.

## 1. Introduction

The Lisfranc joints play an important role in connecting the forefoot and midfoot and maintaining the stability of the arch of the foot [1–3]. With the rapid development of transportation and construction industry in recent years, the incidence of Lisfranc injury has been increasing year by year, and if not treated in time, it will lead to poor walking, pain in the back of the foot, and even disability in severe cases [4–6]. Therefore, it is extremely important to choose a suitable and effective treatment method to treat Lisfranc joint injury. At present, the treatment of Lisfranc joint injuries is mostly through open reduction and internal fixation. Clinically, there are many ways to choose internal fixation, mainly including Kirschner wire internal fixation, hollow screw internal fixation, and steel plate internal fixation [7, 8]. Kirschner wire internal fixation has the advantages of simple operation and low cost, but its stability is poor, and the bone block is very easy to slip [9, 10]. The screw internal fixation effect is good, and it can solve the shortcomings of the poor stability of Kirschner wire fixation, but it is easy to cause damage to the articular cartilage surface and cause traumatic arthritis [11, 12]. The steel plate internal fixation not only has a fixation effect similar to that of screw internal fixation but also avoids damage to the articular surface of the Lisfranc joint to reduce the occurrence of traumatic arthritis [13, 14]. This study aims to explore the curative effect and biomechanical evaluation of three internal fixation methods of Kirschner wire, hollow screw, and steel plate in the treatment of Lisfranc joints injury and to provide corresponding theoretical basis for the choice of clinical internal fixation, in order to improve the efficacy of Lisfranc joint injuries. The specific report is as follows:

## 2. Materials and Methods

### 2.1. Patients

A total of 92 patients with Lisfranc joint injuries admitted to our hospital from March 2017 to September 2019 were selected as the research objects. There were 52 male and 40 female, aged from 26 to 74 years, with an average age of (47.68 ± 10.56) years. The causes of injuries were 19 cases of traffic accidents, 32 cases of sports sprains, 26 cases of injuries from falling from heights, and 15 cases of injuries from heavy objects. Among them, 59 cases were injured in three columns (medial, middle, and lateral), 13 cases were injured in two columns (medial and middle), and 20 cases were injured in two columns (medial and lateral). According to the different methods of internal fixation, the patients were divided into the following three groups: the Kirschner wire group (29 cases), screw group (31 cases), and steel plate group (32 cases). Inclusion criteria: all patients meet the diagnostic criteria for Lisfranc joint injury [15, 16]; anmetabolic bone disease; all of them met the surgical indications; and clinical data were complete. Exclusion criteria: those with severe injury and unable to undergo internal fixation surgery; those with severe coagulation dysfunction; those with rheumatic or gouty arthritis; those with old Lisfranc joint injury; and those with follow-up loss. Comparison of general information of the 3 groups showed no statistically significant difference (*P* < 0.05), and they were comparable, as shown in Table 1.

### 2.2. Treatment Method

When the swelling of the affected foot subsided and wrinkle signs appeared, the surgical treatment was performed with internal spinal anesthesia or general anesthesia. According to the type of Lisfranc joint injury, 1–3 longitudinal incisions on the dorsum of the foot were chosen to protect the dorsal blood vessels, deep peroneal nerve, and cutaneous nerve, stretch the extensor tendon, destroy the interplantarsal and intertarsal ligaments as little as possible, often lift the avulsed bone fragments to reveal the joint, remove the free small fragments in the joint space, fix the bone joint under direct vision with precise repositioning of fine Kirschner pins, and choose Kirschner pins, screws, and microplates for final fixation after satisfactory C-arm machine fluoroscopy. Kirschner wire group: the 1.5 mm Kirschner wire was used to fix the metatarsophalangeal joint through the percutaneously or subcutaneously across the joint in a longitudinal oblique row, and the fine Kirschner wire was pulled out. Screw group: first, a guide needle was taken and driven from the medial cuneiform into the second metatarsal base or from the second metatarsal base into the medial cuneiform. Then, according to the injury of the medial column and the middle column, the guide pin was inserted into the Lisfranc joint or horizontally into the cuneiform. After the C-arm fluoroscopy guide wire was in position, a 3.0 mm hollow screw was chosen to fix the Lisfranc joint along the guide wire, and then, the guide wire and the fine Kirschner wire were removed. Steel plate group: after precise repositioning of the Lisfranc joints, temporary fine Kirschner wires were used for fixation, and the medial column and middle column of the Lisfranc joints were fixed with a plastic arch bridge-like general or locking miniature steel plate, and the fine Kirschner wires were removed. In all cases with outer column injury, the outer column was internally fixed with 1.5 mm Kirschner wire after reduction (as shown in Figure 1).

At the same time, all patients were given prophylactic use of antibiotics, raised limb immobilization, regular dressing change to keep the incision dressing dry, and detumescent drugs to reduce foot swelling, the drainage tube is generally placed for 1–2 days after removal, and stitches can be removed after 2 weeks. Early rehabilitation training was given according to the patient's recovery, and attention should be paid to avoid internal fixation fracture during training.

### 2.3. Observation Index

The patients were followed up for 6 months after the operation to observe their complications, and their foot function was evaluated according to the American Orthopaedic Foot and Ankle Society (AOFAS) [17] scoring system. 90 or greater is considered excellent, 75–89 is good, 50–74 is fair, and less than 50 is bad, excellent and good rate = (excellent + good)/total number of cases ×100%. Before operation and during follow-up, the pain scoring visual analogue scoring method (VAS) was used to evaluate the pain. Different fixation models were established according to different fixation methods: point reduction forceps were used to fix the medial cuneiform and the second metatarsal, and Kirschner wires, screws, and the steel plates were used to fix the medial cuneiform and the second metatarsal, respectively. The Kirschner wire group and the screw group applied a maximum axial pressure of 350 N to the tip of the specimen at a speed of 10 N/s, the steel plate group applied a maximum axial pressure of 600 N, and the maximum load is maintained for 5 seconds. We used this to calculate the displacement change between the medial cuneiform bone and the second metatarsal base. A maximum of 50 N abduction force was applied to the three groups at a speed of 2 N/s, and the maximum load was maintained for 5 seconds before the end, to calculate the displacement change between the medial cuneiform bone and the second metatarsal base. Three groups of continuous testing were conducted for 3 cycles, with an interval of 3 min between each cycle. Middle column injury model: the injury model of the middle column of the metatarsal tarsal joint was established by disconnecting the second and third metatarsal tarsus joints of the middle column of the metatarsal tarsus joint and the dorsal ligament, interosseous ligament, and metatarsal ligament connected with the surrounding middle column. It was planned to use the compressive stress experiment to compare the biomechanics of the abovementioned three groups of different methods of internal fixation; that is, we performed a pressure test on the middle column of the Lisfranc joint after internal fixation and recorded the peak pressure data after the middle column was completely collapsed.

### 2.4. Statistical Method

The results of this experiment were statistically analyzed by SPSS 20.0 (SPSS Co., Ltd., Chicago, USA). Count data were expressed by (rate), and the chi-square test was used for their comparison between groups. Measurement data were expressed by (mean ± standard deviation), and the *t*-test was used for their comparison between groups. *P* < 0.05 indicates that the difference is statistically significant.

## 3. Results

### 3.1. Comparison of Joint Recovery of Patients in Each Group

In the Kirschner wire group, 6 cases were excellent, 10 cases were good, 9 cases were fair, and 4 cases were poor, with an excellent and good rate of 55.17% (16/29). In the screw group, 9 cases were excellent, 12 cases were good, 7 cases were fair, and 3 cases were poor, with an excellent and good rate of 67.74% (21/31). In the steel plate group, 10 cases were excellent, 16 cases were good, 5 cases were fair, and 1 case was poor, with an excellent and good rate of 81.25% (26/32). The excellent and good rate of the steel plate group was higher than that of the Kirschner wire group and screw group (*P* < 0.05), as shown in Figure 2.

### 3.2. Comparison of Pain Conditions in Each Group

During the follow-up at 1, 3, and 6 months after the operation, the VAS scores of the steel plate group and screw group were significantly lower than those of the Kirschner wire group, and the steel plate group was significantly lower than the screw group (*P* < 0.05), as shown in Figure 3.

### 3.3. Postoperative Complications in Each Group of Patients

In the Kirschner wire group, there were 2 cases of traumatic arthritis, 2 cases of incision infection, 2 cases of foot arch collapse, 1 case of internal fixation loosening, and 1 case of joint stiffness, and the total incidence of complications was 27.59% (8/29). In the screw group, there was 1 case of traumatic arthritis, 1 case of incision infection, 2 cases of foot arch collapse, 1 case of internal fixation loosening, and 1 case of joint stiffness, and the total incidence of complications was 19.35% (6/31). In the steel plate group, there was 1 case of traumatic arthritis, 1 case of incision infection, and 1 case of joint stiffness, and the total incidence of complications was 9.38% (3/32). The total incidence of postoperative complications in the steel plate group was lower than that of the Kirschner wire group and the screw group (*P* < 0.05), as shown in Figure 4.

### 3.4. Comparison of Biomechanical Indexes in Each Group of Patients

The axial displacement and abduction displacement of the steel plate group and the screw group were smaller than those of the Kirschner wire group, and the peak pressure was higher than that of the Kirschner wire group (*P* < 0.05). The axial displacement and abduction displacement of the steel plate group were smaller than those of the screw group, and the peak pressure was higher than that of the screw group (*P* < 0.05), as shown in Figure 5.

## 4. Discussion

The generalized Lisfranc joints also include intermetatarsal joints and intercuneiform joints, which are called Lisfranc joint complexes [18]. Sands [19] proposed the three-column theory of the Lisfranc joint based on the anatomical basis: the medial column is composed of the first cuneiform and the base of the first metatarsal; the middle column is composed of the second and third metatarsals and the second and third metatarsal bases. Among them, the second metatarsal bone and the third cuneiform bone form a tenon-like structure, which is an important part of the stability of the Lisfranc joint. The lateral column includes the joint in front of the cuboid bone and the base of the fourth and fifth metatarsals. At the same time, the Lisfranc joint participates in the formation of the medial longitudinal arch (medial and intermediate column), lateral longitudinal arch (lateral column), and transverse arch (Lisfranc complex), which play an important role in the weight-bearing and walking cycle. Lisfranc joint injury often manifests as simple Lisfranc joint dislocation or fracture dislocation. With the rapid development of transportation and construction industries in recent years, the incidence of Lisfranc injury is increasing year by year [20–23]. Due to the complex anatomical structure of the Lisfranc joint and various injury mechanisms, it is easy to be misdiagnosed in clinical diagnosis, and the misdiagnosis rate can be as high as 20%. The Lisfranc joint is an important part of the arch of the foot. Once injured, the transverse and longitudinal arch of the foot will often be destroyed. If the treatment is not timely or standardized, the patient will have discomfort in walking, chronic pain, and even forefoot deformity, traumatic arthritis, and other complications, which will have a serious impact on the weight bearing and function of the foot [24–26]. At present, a large number of studies have shown that open reduction and internal fixation can achieve good clinical efficacy in the treatment of medial column injury of metatarsal joint. There are various internal fixation methods in clinical practice, including Kirschner wire internal fixation, hollow screw internal fixation, and plate internal fixation. At present, the controversy in the treatment of Lisfranc injury lies in the choice of internal fixation materials. Therefore, it is of great significance to explore the efficacy of different internal fixation materials in the treatment of tarsal injury. Our hospital has a wealth of clinical experience in the treatment of Lisfranc joint injuries. This study summarizes our physicians' years of experience in the treatment of Lisfranc joint injuries to provide a certain reference for clinical applications.

The results of this study showed that the excellent and good rate of the steel plate group (81.25%) was higher than that of the Kirschner wire group (55.17%) and screw group (67.74%). During the 1-, 3-, and 6-month follow-up after the operation, the VAS scores of the steel plate group and the screw group were significantly lower than those of the Kirschner wire group, and the VAS score of the steel plate group was significantly lower than that of the screw group. The reason for this is that the strength of the internal fixation of the Kirschner wire is not high, and it was easy to break leading to instability of fixation and slippage of the bone block, which affects the functional recovery of the patient's foot. The screw internal fixation can provide better fixation strength than the Kirschner wires. However, during postoperative functional exercises, the concentrated load stress of the screw is relatively large, which may easily lead to broken nails and change the reset position, affecting postoperative recovery. The steel plate internal fixation can not only provide reliable fixation but also carry most of the load stress, and it is easier to remove than screws after fracture, which is conducive to the recovery of joint function [5, 27, 28]. The results of the study showed that the total incidence of postoperative complications in the steel plate group was lower than that of the Kirschner wire group and the screw group. This shows that there are fewer complications after the steel plate internal fixation. The reason is that the strength of Kirschner wire is not high and the tail of the needle is left outside the skin, which cannot resist the external force of the middle foot, leading to fracture prone to slip, unstable fixation, and loss of reduction. Compared with Kirschner wire, screw can provide greater fixation strength and pressure effect, so patients are less likely to have fixation loosening after surgery. At the same time, open reduction can achieve accurate joint alignment. However, for joints with greater range of motion, screw concentration has greater load stress, resulting in increased chance of screw breakage. As screw joint surface grinding is unable to deal with the damage, the steel plate fixation can have good fixation effect, high elasticity, and fix to the bone surface tightly, will not cause further damage to joint surface, can well adapt to joint bending stress, reducing the joint degenerative diseases, mostly carries load stress at the same time, and also does not easily break.

The biomechanical results of this study showed that the axial displacement and abduction displacement of the steel plate group and the screw group were smaller than those of the Kirschner wire group, and the peak pressure was higher than that of the Kirschner wire group. The axial displacement and abduction displacement of the steel plate group were smaller than those of the screw group, and the peak pressure was higher than that of the screw group. It showed that steel plate had more advantages in bearing pressure than screws and Kirschner wires. The Kirschner wire is thin and round, which is used for the middle column and the medial column that need to be stabilized. It has poor compression resistance and weak fixation; especially in patients with osteoporosis, the fixation strength is insufficient. The Kirschner wires are also often used for elastic fixation or open injury of the lateral column, poor skin and soft tissue conditions, and temporary treatment of compound injuries in emergency. The screw has a relatively stable connection and fixation function, but its pressing arm is small and the force is concentrated. When the pressure is large, it is easy to cause the screw to loosen, causing the fracture end to shift or the screw to break, and the articular cartilage surface will be further damaged after joint fixation and repeated nail penetration, which may increase the probability of traumatic arthritis. However, the use of an ordinary or locked microsteel plate of plastic arch bridge for transarticular internal fixation of the middle column and the inner column can well maintain the normal physiological radian of the longitudinal arch of the foot. Compared with the screw internal fixation, the acting pressure arm is larger, and the force is uniform and the bearing capacity is good, which has a better stability effect [6, 29, 30]. Through repeated surgical operations and mutual learning and discussion after surgery, our physicians had summarized some experiences. We believe that the key to the treatment of Lisfranc joint injury is to accurately reset the joint and the establishment an effective fixation, so that the anatomical relationship of the body's transverse arch can be restored, so as to complete its gravity conduction and improve the quality of life of patients.

## 5. Conclusions

Compared with Kirschner wire and screw internal fixation, the use of shaped arch bridge-type microsteel plate internal fixation for the treatment of metatarsotarsal joint injury patients showed better foot function recovery, fewer complications, and more reliable biomechanical strength.

## Figures and Tables

**Figure 1:** Diagram of the surgical procedure: (a) Kirschner wire group (preoperative); (b) Kirschner wire group (postoperative); (c) screw group (preoperative); (d) screw group (postoperative); (e) steel plate group (preoperative); and (f) steel plate group (postoperative).

**Figure 2:** Comparison of joint recovery of patients in 3 groups. *Note*. Compared with the Kirschner wire group, ^*∗*^*P* < 0.05; compared with the screw group, ^#^*P* < 0.05.

**Figure 3:** Comparison of pain conditions of patients in 3 groups. *Note*. Compared with the Kirschner wire group, ^*∗*^*P* < 0.05; compared with the screw group, ^#^*P* < 0.05.

**Figure 4:** Postoperative complications of patients in 3 groups. *Note*. Compared with the Kirschner wire group, ^*∗*^*P* < 0.05; compared with the screw group, ^#^*P* < 0.05.

**Figure 5:** Comparison of biomechanical indexes of patients in 3 groups: (a) Comparison of the axial displacement of the 3 groups of patients; (b) comparison of the abduction displacement of 3 groups of patients; (c) comparison of the peak pressure of 3 groups of patients. *Note*. Compared with the Kirschner wire group, ^*∗*^*P* < 0.05; compared with the screw group, ^#^*P* < 0.05.

**Table 1:** Comparison of 3 groups of general information.

Groups	n	Age (years)	Gender		Cause of injury			
			Male	Female	Traffic accidents	Sports sprains	Fall from height	Heavy object crush
Kirschner wire group	29	47.46 ± 10.93	17	12	6	9	9	7
Screw group	31	47.64 ± 10.65	16	15	5	12	6	4
Steel plate group	32	47.92 ± 10.08	19	13	7	11	11	4
*F/χ* ^2^		0.015	0.462		2.854			
*P*		0.985	0.794		0.827			

## Data Availability

The data can be obtained from the author upon reasonable request.
